RETRACTED

# QoS-Aware Smart Phone-Based User Tracking Application to Prevent Outbreak of COVID-19 in Saudi Arabia

**DOI:** 10.1155/2022/2273910

**Published:** 2022-04-11

**Authors:** Arwa Mashat, Aliaa M. Alabdali

**Affiliations:** Faculty of Computing & Information Technology, King Abdulaziz University, P.O. Box 344, Rabigh 21911, Saudi Arabia

## Abstract

Diverse variants of COVID-19 are repeatedly making everyday living unstable. In reality, the conclusive retort of this highly contagious virus still is in incognito mode. The health experts' primary guideline on the possible prevention of this disease outbreak, including a list of restrictions and confinements, is insufficient in case of any public congregation. As a result, the demand for precise and upgraded real-time COVID-19 tracking and prevention-based applications increases. However, most of the existing android-based applications face a lack of data security and reliability that cannot satisfy the additional quality of service (QoS) requirements. This paper proposes an easy-to-operate android-based multifunctional application to track individuals' health situations, allow uploading scanning report by the authorized organization like universities, mosques, school, and hospitals and helps the users to maintain guidelines via manageable steps. This article offers a three-layered QoS aware service-oriented task scheduling model upon multitasking android-based frontend focusing the cognitive-based AI applications in healthcare with a continual learning paradigm. Designed model is competent to optimize heterogeneous service scheduling and can minimize data delivery time, as well as the resource cost.

## 1. Introduction

Like many countries worldwide, massive numbers of people in the Kingdom of Saudi Arabia (KSA) are losing their income due to the close of numerous companies and businesses, in an attempt to stop the spread of COVID-19 [1]. The Saudi Health Ministry spokesman confirms that because of the new COVID-19 variant, Saudi Arabia are witnessing a jump in COVID-19 cases. In contrast, the Saudi Ministry of Commerce spokesman notified the required measurement of commercial businesses to control the spread of COVID-19. Considering the vulnerable financial situation and the high risk of the new variant, the government has stressed priority-based reopening of public sectors as soon as receiving necessary vaccine doses. We propose a multitasking connective android-based interface to allow the public organization to scan individuals at their entry points. And to upload the latest report to the Ministry of Health databases against the visitors' National or Iqama ID, using Hemayah application. The primary objectives of the suggested approach are as follows.

- Technical help: to allow companies and sectors to scan individuals in a group and update their current health status through an easy-to-use android interface.
- Contactless approval: without physical contacts like a hard copy of a report or mobile phone handover. Permission to enter an organization, depending upon the most recent physical condition.
- Time to time test: the person does not have to go through testing before going to a public gathering. Still, they have to follow the basic guidelines as they enter a public place.
- Regular scanning and data update: a person does not have to go physically to a medical center for the latest physical report and upload it to the Ministry of Health database if an organization has permission to scan individuals at the entrance.
- Updated news and information: to fight against the new variants, the Hemayah provides suggestions by the health experts, including news, analyses curves, and statistics.
- Worldwide acceptance: the chosen authorized organizations will be connected to the same network. Therefore, visitors could avoid the lengthy queues at border checkpoints.
- System to system connectivity: the individual does not need to connect every time to the databases. The authorized server can access the data of a person with their due permission makes possible minimum Internet data and bandwidth usage at a public gathering place with the help of cognitive computing.

RETRACTED

The model has explored a near-optimal service at the application layer by making user data metrics through detailed observation of each tracking component. The QoS manager deals with various network traffic difficulties at the network layer to schedule heterogeneous service demands. The model ensures information accuracy at the database layer and works on adaptability factors for assorted service demands.

## 2. Related Work

Smartphone-based applications are connected with the cloud databases/remote databases and provide real-time updated information. The government cites provide authenticated pubic data to notify the citizens regarding the latest news.

Saudi Arabia's official health ministry web platform against web page provides a home button with other valuable sources like the interactive map, awareness, available e-services, media centers, and open health-related public data. In particular, the data option directs to the open data portal, from where any user can avail COVID-19 statistics, open data library, help, and proposals, including particular usage policies. To the directed COVID-19 statistics e-platform web page (https://covid19.moh.gov.sa/), the latest update about the country's new COVID-19 cases, critical cases, recovered number of cases, deaths, and few interactive maps/graphs in English and Arabic languages are being provided. Smartphone users can download a similar interactive platform from the Google application center. The Kingdom of Saudi Arabia Ministry of Health (MOH) certified applications for smart phone users are Sehhaty, Mawid, Seha, Tawakkalna, Tabaud, Health Volunteering Application' (HVA), Eshara, Qareboon, MOH Formulary App, Mawared, etc [1].

RETRACTED

Android-based application Sehhaty helps individuals in KSA with several assorted health-related assistance. One can avail COVID-19 testing and dependent service, e-prescription, health consultancy, biomarkers, sick leave, primary level of disease prevention and control, including school screening. Using the E-Appointment App Mawid, patients are suggested nearby hospital services, as well as referred doctor's appointments could be made via a seamless track offered by this application. Several technologies proposed in [2, 3] do the same. Another E-health application Seha has a personal assistant service and can connect with MOH's specialists through chatting and audio and video calls. It also sustains artificial intelligence-based assistants for customized medical consultancy and health tips. The audiovisual way helps maintain a better healthy environment in the home. It also registers the users' feedback at the end of the service completion. Similar MOH services are facilitated to the hearing impaired and deaf people through the Eshara application. This android-based application supports sign language and provides medical consultancy, doctors' appointments, and other needed support.

Android-based application Tawakkalna helps to verify own health condition through colored codes. Using this application, the user can report any violation regarding health measurements and infected cases in a public gathering. Subsequently, it helps to split the chain of infection.

Apart from the assistant applications, the Tabaud has been designed to track COVID-19 spread. If the user of Tabaud contacted any COVID-19 confirmed patient in the last few days, it makes cautious of that. Any of the confirmed cases detected by this app sends an immediate proactive notification to its user to break the infection chain. It maintains its user's data confidentiality and decides from the observed data of the last fourteen days. If the prediction of the application and the user confirmation match, then it sends the proactive notification to its other users. The Health Volunteering Application has been designed to connect all the willing users for volunteering works in this pandemic. It allows the volunteers to find a job that matches their skills and fields. The user could observe their achievements through their personal account. One can connect with group volunteering and social activities via community building on this application.

RETRACTED

During this pandemic, mental health was also affected due to job loss and long-term isolation. MOH encourages android-based applications such as Qareboon, which offers text-based mental counselling directed by specialists. One could find an integrated library of knowledge on cognitive healthiness and most delinquent methods, like info graphics, text materials, and audiovisual content.

There is another android-based application called Mawared to help contactless and hassle-free communication between the staff of an enterprise. The staff can apply for sick leave, casual leave, or annual leave via this application. The application has been designed for MOH's staff and helps them submit their assignments, office resumption, etc into the office channel. Apart from these, other android apps available mostly are based on the following features [4–6].

- Official platforms (with websites and other connected databases, sources of information) for daily updates and tracks [7, 8]
- Near-by-you COVID-19 cases indicator apps [9]
- Corona-Warn-Apps focus on reminding its users about the health experts' primary health precautions and guidelines using ML-based learning [10–13]
- Heat map-based apps to update gathering and population velocity in real-time [14]
- Individual data uploading, storing applications help to display when needed at official checking points [15, 16]

## 3. Problem Statement

To reduce the consequences of the pandemic is needed to return the systematic life as the outbreak has drastically affected the economy of KSA. Primary guideline on the possible prevention of this disease outbreak includes a list of restrictions and confinements [17–19]. Many android-based apps have been developed to remind these restrictions to maintain health guidelines. Everyone should maintain the safety guidelines suggested by the health experts; however, these are insufficient in any public congregation. As a result, the demand for precise and upgraded real-time COVID-19 tracking and prevention-based applications increases [20–22]. Multitasking apps support daily updates, visiting places tracking, physical symptoms checking (using Q&A procedure), report downloading, and others. Subsequently, the existing android-based applications lack data security and reliability, consumes more data, resultant request overlapping into public places; unable to satisfy the additional quality of service (QoS) requirements [17, 23]. We concentrated on the current two situations/problems: individuals' entry into public gatherings and border checkpoints with the help of cognitive-based AI application to the backend. We concentrated on the current two situations/problems, shows in Figure 1: individuals' entry into public gatherings and border checkpoints with the help of cognitive-based AI application to the backend.

RETRACTED

**Case 1 .**

Elaborated into Figure 1(a); Standing in a queue and waiting to show their updated COVID-19 related report; like a student in front of a university or a group of individuals in front of a mosque. Every individual has to show their latest COVID-19 negative report and vaccinated certificates to participating in the restricted gathering. Whether it is a hardcopy (a piece of paper) or a softcopy (downloaded/ stored data) from a phone database, it needs to be handed over and subsequently causes disease transfer. Another point is that if a person is found to be a COVID-19 positive at the entrance of that association, there is no provision to update their latest condition in traditional Android-based applications. In this gathering, numerous authorized searches (OTP-based authorization for login) for the latest COVID-19 report from govt./private site, random searches for the latest news update; using similar Android applications is realistic. As a result, similar service requests by the persons in the queue/ group arise a high chance of service failure. Similar service requests also cause higher data consumption due to high traffic. More costing and poor battery life are also involved as a passive result.

In this case, the association/sector, where the person wants to get entry, and the report provider authorization/administrator has a different application website and application server (Within the same country). Therefore, we can transfer soul authority to the particular association/sector to scan every incomer, verify their given report/information from direct to that administrative website, and update the individual's latest health clearance without any human contact. Hemayah offers this exact digital platform with AI learning [24, 25] and helps to reduce document hardcopy/phone handover during entry into public assemblages.

**Case 2 .**

Elaborated into Figure 1(b); Standing in a queue and waiting to show their updated COVID-19 related report in a country-checkpoint, arriving from a different country.

Here, the distinct authenticated organizations belong to different countries. Authorized organization/sector administrator belongs to KSA. Similarly, there is no authorization to access/exchange data to update the latest about the newly arrived person to the global database except the Local DB check for previously stored data.

RETRACTED

Therefore, we can transfer soul authority to the particular association/sector to scan every incomer, verify their given report/information directly to that administrative website, and update the individual's latest health clearance without any human contact. The application also provides a database in which the authorities in the Kingdom of Saudi Arabia allow specific lab centers to be accredited worldwide through embassies to enter reports of the person's condition, whether he is infected with the disease or not. The data of peoples' status is recorded in the database according to the passport numbers. At the point of entry to the Kingdom, the passport employee can view the report of the inside crossborder using an indifferent platform. This feature prevents paper reports that may be subject to fraud. It also guarantees the reliability of the result, as the country will not approve the reports issued by the predetermined laboratories. Both of the solutions have been portrayed into Figure 2.

## 4. Proposed Solution

The application offers several contributions that have not been offered before, namely:

- The authorities can directly verify the status of people through their stored status in the database.
- The application allows the authorities to scan the incoming people in one group, and in the event that there is a confirmed case within the group, the application saves the contact information and turns their statuses into (contacted) to alert the health authorities.
- To allow authorities to scan so that the person scanning guarantees the validity of the data provided to him not as in Tawkkalna or Tabaud app, where the status is only presented to the user. While in Hemayah, the person entering the data is the one who belongs to the authorities and not the person to whom the data is to be presented.
- The application also provides a database in which the authorities in the Kingdom of Saudi Arabia allow certain lab centers to be accredited all over the world through embassies, to enter reports of the person's condition whether he is infected with the disease or not.
- The data of peoples' status is recorded in the database according to the passport numbers, and at the point of entry to the Kingdom, the passport employee can view the report of the inside crossborder.
- Hemayah application is smart and easy to control; powered by cognitive-based artificial intelligent backend which analyze response from patients to establish cure efficiency.

This feature prevents paper reports that may be subject to fraud. It also guarantees the reliability of the result, as the reports issued by the predetermined laboratories will not be approved by the country. To model a composite architecture of an android-based application, at first we need to point out the three layers in top to bottom approach, as follows:

- Decision making at application layer
- Decision making at network layer
- Decision making at database layer

QoS parameters in our proposed COVID-19- foundation model is basically depend upon some real time network factors like available bandwidth, network layer capacity, demands and some defined factors like subject of authorization, system-to-system data sharing, recapitulation of data etc. We have discussed all these possible QoS variables separated layer based with suitable definitions and formulas for real-time adaptive multifunctional android application, called Hemayah.

RETRACTED

### 4.1. Service Metric at Web-Service or Application Layer

The android application layer is also known as the web service layer, shows in Figure 3. The android application layer is also known as the web service layer. The application-based subscribers' end or front end is connected with network operators. Depending upon the service-layer agreement, the Hemayah application offers the following:

- Login activity page: individual-based, organization-based
- Information panel: basic information like user's National or Iqama ID, phone number, individual's or company e-mail id
- Navigation bar: with list of facilities, visualization of personal database
- Location-based update: last visiting place and contacted person list
- Scanning data upload: by authorized organization, country border side checkpoint admin etc.

In this layer which service parameters has considered to build our proposed model are following:

1. )Service Charge *C*(*β*)*:* service charge typically represents the service supplying cost to the network operator. It also refers to the service subscribing price against quality of service matrices. A service charge for unit-based data provision is usually invariant or specified by service operators.
2. Service Time *I*(*β*)*:* the service operator takes the overall time; from the time of a registered query selection to the time to compile and fulfill that service request is called service time. This request completion time typically depends upon the network traffic, resource/database finding, process capability of the service manager, request compilation by the specific data server, authorization checking, and other network-related factors. The time of service request completion can be measured by:
3. *E*(*I*(*β*))=(*πρ*_*k*_)/((1 − *π*)^2^*ε*+1/*μ*); against a numbers of application nodes *k*, for *N*/*N*/*k* queuing model.
4. Service Load *L*(*β*)*:* a service provider does not encounter identical submissions at any time. Service utilization measures the service load at a specific time by its authorized subscribers. The equation can ideally calculate it: *L*(*β*)=*εμ*. When the service requests arrive at a rate of *ε*, and the request-to-response rate of the service operator is *μ*.
5. Service Reliability Re(*β*)*:* to match the expected service rate and service consistency of the maximum subscriber is counted as the reliability of the service provider. It is also measured by the probable failure of service request completion on the application end, is denoted as Re(*β*), a hit and miss counter, measured by ∑_*k*=1_^*N*^*x*_*i*_/*n* and *D*.

RETRACTED

Service Reputation Rp(*β*): The subscriber-level prominence is called service reputation. A better quality of experienced uplifts the reputation of an android application at the user level. Increased trust levels promote the application to other groups of users.

- QoS of App-Service Architecture: QoS rarely focuses on another term called quality of experience (QoE). A different between the expected service and the actual experience makes them different in character. Most of the time service provider fails to touch the expectation line of the consumers due to the high conspiracy nature of overlapped networks. Our aim is to design alive-QoS manager module in between task queue and allocated service as a decision making unit for near optimized service scheduling. The module is communicating between single point scanning point and application layer so that it can be defined as QoE metrics provider/monitoring module. At this point if assumed QoS metric results are denoted by A and the confidence level to update the resultant metrics is *γ*, depending upon Ε(*A*) and *D*(*A*), the interval of confidence will be defined as $\left(E\left(A\right)\right.-\sqrt{\left(D\left(A\right)/\left(1-\gamma \right)\right)}$, $\left(E\left(A\right)\right.+\sqrt{\left(D\left(A\right)/\left(1-\gamma \right)\right)}$. The recent scanning report is stored against an individual.
- Service Quality Measurement and Task Model*:* let us assume (*T*, *X*, *P*, *R*) is a four-tuple decision making process or DMP model which is consisting of *T*, i.e. denotes the set of states, *X*: the set of action (as the proposed application offers multi-funtional front end). Probability function *P* is described as (*P* : ∈[0,1]), the state changes from service request off mode to on mode and vice versa. And the last tuple *R*(*t*, *x*) denotes the reward function of an action which is able to change the previous status from (*t*) So that *R* : *T* × *X*⟶*R*.

Proposed model depends upon the quality of a policy, which is measured by the expected sum of the service rewards. To ensure the finite up gradation of *E*(*R*), some of the time it may varies and discount may be offered by the providers. *F*^*ρ*^(*t*) represents the sequence of states and can be achieved within the policy *ρ* from the equation (1).

(1) $$\begin{array}{c} F^{\rho }\left(T\right)=\underset{x\in X}{\arg\max}\left(R\left(t,x\right)+\alpha \sum_{t^{\alpha }\in T}p\left(t,x,t^{\prime }\right)F^{\gamma }\left(t\right)\right). \end{array}$$

We have another equation:

(2) $$\begin{array}{c} R\left(t,x\right)=\sum_{t^{\prime }\in T}R\left(t,x\right)\times p\left(t,x,t^{\prime }\right). \end{array}$$

The optimal policy can be obtained from above equations; further optimized form is shown in equation (3).

(3) $$\begin{array}{c} F\left(T\right)=\underset{x\in X}{\max}\left(R\left(x,t\right)+\alpha \sum_{t^{\prime }\in T}p\left(t,x,t^{\prime }\right)F^{\gamma }\left(t\right)\right). \end{array}$$

Optimal policy value of *F*_*k*_ can be obtained at the point *k*⟶*∞*. Let a user is consuming an Hemayah service at the time instant *i* and the state is defined with three tuple (*i*, *l*, *e*) where *i* ∈ {*i*_1_, *i*_2_,…, *i*_*I*_} is the measurement variable used to measure the previous time-state *e* is the consumed amount of power. If *t*_*i*_=(*i*_*j*_, *l*_*j*_, *e*_*j*_) and *t*_*j*_=(*i*_*k*_, *l*_*k*_, *e*_*k*_) are the two transition states before and after an action of *x* ∈ *X*, then the transaction probability is *p*(*t*_*j*_, *x*, *t*_*k*_), can be modified for the various available probabilities of bandwidth, energy consumption and state model as *p*_bw_(bw_*j*_, bw_*k*_), *p*_*e*_(*e*_*j*_, *e*_*k*_), *p*_*i*_(*i*_*j*_, *i*_*k*_).

RETRACTED

Where

(4) $$\begin{array}{c} p_{I}\left(i_{j},i_{k}\right)=\left\{\begin{array}{cc} 1, & \text{if }j=k=1,\\ -1, & \text{if }k=j+1,\\ 0, & \text{if otherwise,} \end{array}\right. \end{array}$$

is the definition of the state model with the changes of bandwidth is shown in equation (5).

(5) $$\begin{array}{c} p_{\text{BW}}\left({\text{bw}}_{j},{\text{bw}}_{k}\right)=\left\{\begin{array}{c} p_{\text{BW}}^{\text{same}}\text{,}\;\text{if }i=k;\\ 2p_{\text{BW}}^{\text{change}}\text{,}\;\text{if }j=\text{BW},j=2\text{ BW};\\ p_{\text{BW}}^{\text{change}}\text{,}\;\text{if }\left|j-k\right|=1;\\ 0,\;\text{otherwise,} \end{array}\right., \end{array}$$

and the probable consumption of energy can be modeled as per equation (6), for the action occurrence *x* ∈ *X*.

(6) $$\begin{array}{c} p_{E}\left(e_{j},e_{k}\right)=\left\{\begin{array}{cc} 1\left(a\right), & \text{if }j=E,\\ p_{e}, & \text{if }j=BW,\\ 1-p_{e}^{\left(a\right)}, & \text{if }j+1=k,\\ 0, & \text{otherwise.} \end{array}\right. \end{array}$$

In the term of the reward function we have to depend upon the information about available bandwidth which is only can be reported by the edge nodes. Here, we use equation (7) to sum up the reliability model of our proposed architecture:

(7) $$\begin{array}{c} R\left(\left(i,y,e\right),x\right)=\left\{\begin{array}{cc} -R^{\text{powerout}}, & \text{if }e=E,i<I;\\ k_{R}.x.y, & \text{otherwise.} \end{array}\right. \end{array}$$

Where *k*_*R*_ is the proportionality constant? Equation (6) can be easily solved if it is assumed that each edge node runs for each single task for once for single consumed service. This probable condition can be initialized from a state defined as *F*_0_^(*t*)^ and further can be updated for an iteration of *k* > 0, shown like equation (8).

(8) $$\begin{array}{c} F_{k}\left(T\right)=\underset{x\in X}{\max}\left(R\left(t,x\right)+\alpha \sum_{t^{\prime }\in T}p\left(t,x,t^{\prime }\right)F_{k-1}^{\left(t\right)}\right). \end{array}$$

Here, we proposed single point hassle-free easy-to-use android-based application. By entering the visitor's National or Iqama ID, Hemayah allows users to check the status of anyone in front of them from their mobile phones without the need to use the visitor's phone. The request is here made by the entry point of that particular organization using the visitor ID. The communication is system-to-system.

RETRACTED

Algorithm 1 represents the step by step view for Iterative Model of QoS aware Hemaya's database selection towards Cases 1 and 2 solutions.

And the reward function *R*(*t*, *x*) then starts to follow the further rule of equation (9).

(9) $$\begin{array}{c} R\left(t,x\right)=\sum_{t^{\prime }\in T}R\left(t,x,t^{\prime }\right)p\left(t,x,t^{\prime }\right). \end{array}$$

### 4.2. Decision Making in the Network Layer

Service selection decision directly depends upon the network traffic into the network layer, which can be gained for two different types of services. Determined by the probable service compilation time, i.e. delay or jitter sensitive services. [Ex. Some real-time execution based services]. Another is *z* Based services, where *z* stands for some non-predetermined network variables like location, peer-to-peer applications. Application page/node needs a minimum provisional connectivity rate Rate_min_^(*i*)^ for *i*=1,2,…*k*. Where the optimal function of service selection looks like equation (10).

(10) $$\begin{array}{c} F_{k}\left(t\right)=\sum_{x\in X}p\left(t,x,t^{\prime }\right)\left[R\left(t,x\right)+\alpha F_{k-1}\left(t^{\prime }\right)\right]. \end{array}$$

The optimal policy function for the multifunctional Hemayah services *β* is defined as:

(11) $$\begin{array}{c} f^{*}\left(t\right)=\left\{f^{*}\left(t_{1}\right),f^{*}\left(t_{2}\right),\ldots ,f^{*}\left(t_{N}\right)\right\}. \end{array}$$

For a standard model of QoS for three-layered network we need an optimal proportional fairness of provided service. That means each individual application end should be offered equal resources for each probable transmission. QoS manager should distribute the available services among the application subscribers who are paying equal cost to achieve same offered services. As Hemayah service has a layered architecture, we assume, the *M* numbers of application nodes are belonging to the application layer having mess connection with the *N* numbers of layer-2 operators of the network layer. At a time instant *i*, for a connectivity between *k* nodes of sensing layer and *j* nodes of network layer, total consumed power and bandwidth are denoted by *E*_kj_ and BW_kj_. Then at the node *M*_*k*_, calculated throughput is:

(12) $$\begin{array}{c} r_{k}=\sum_{j=1}^{N}\left(1-\eta_{kj}\right).\delta_{j}.{\text{bw}}_{\text{kj}}\log_{2}\left(1+\frac{g_{\text{kj}}.e_{\text{kj}}}{a_{\text{kj}}}\right). \end{array}$$

Where *k*=1,2,…, *M* and the average bit error rate (BER) of the connectivity (*k*, *j*) is denoted by *η*_kj_. A node says *m*_*k*_, belongs to the edge layer can be guaranteed the bandwidth connectivity at the time instant *i* to access all *t*_*j*_, *a*_kj_ in network layer must having a system efficiency *δ*_*k*_ with channel gain *g*_kj_ and transmission power:

(13) $$\begin{array}{c} e_{\text{kj}},\text{for }r_{j}\geq {\text{Rate}}_{\min}\left(k\right). \end{array}$$

To maximize the QoS of the proposed network, the system capacity should be modified, which can be modeled as following:

(14a) $$\begin{array}{c} \max\text{ Rate}\left(a,e\right)=\max\sum_{j}^{N}\sum_{k}^{M}\left(1-\eta_{kj}\right).\delta_{k}.a_{kj}.\;\log_{2}\left(1+\frac{g_{\text{kj}}e_{\text{kj}}}{a_{\text{kj}}}\right), \end{array}$$

(14b) $$\begin{array}{c} \text{Such that }a_{\text{kj}}\leq A_{j}\forall j, \end{array}$$

(14c) $$\begin{array}{c} \text{And }e_{\text{kj}}\leq E_{k}\forall k. \end{array}$$

Applying convex optimization method, equations (14a)–(14c) can be easily solved. Available bandwidth of both authorized servers can be shared where *E*_*k*_ the maximum consumed power at node is *m*_*k*_ and service manager allocated bandwidth at node *n*_*j*_ is BW_*j*_.

RETRACTED

### 4.3. Decision Making at the Database Layer

The android-based application using local database has some typical natures like limited resource, autonomous personality, with specific-data-collection capacity and susceptibility. Low power, small life time, limited resource, autonomous and randomly deployment of the mobile phones damage the efficiency of any networks, which are sensitively designed for sum specific applications within a specific operation area.

As mentioned, to nourish the Quality of Experience crisis we have to consider these following factors while design the QoS metrics for explicit database connectivity layer.

- Accuracy measurement of the information which is different from the traditional wireless network as authorized data stored in authorized web server are suffering from information comprise illness
- Consumed energy measurement which is also important because application nodes (mobile phone) of the network are typically consumed more data when similar service requests overlapped in a situation like public gathering
- Coverage calculation which is also should be considered to make the whole connectivity network adaptable, energy efficient and load should be optimized with minimum number of connectivity links

In this paper, we emphasize the following matters, accuracy of the collected data, energy efficiency, network coverage and adaptability increases. In web application layer, the performance metrics of QoS extensively fluctuate from the regular android-based network and the input metrics should consider some factors Accuracy Measurement of the Information, latest scanning report available etc.

Information accuracy of measured data can be quantified through some measurements. The higher probability to match the data with the subscription level of user ID (authorization ID of the organization worldwide), the data ensures higher information accuracy. Let *a* ∈ *A*(*β*) is a random data variable passing through the service channel *β* have *N* numbers of status, generated by the *k*^th^ application node. If *θ* denoting the probability of wrong information acquisition then the probability of information accuracy at the subscribers end can be measured by the following equation:

(15) $$\begin{array}{c} p\left(a\right)=1-p\left(a^{\prime }\right). \end{array}$$

Here, *p*(*a*′) is the probability of damaged information delivery due to path-loss exponent and other network-traffic factors. Therefore,

(16) $$\begin{array}{c} p\left(a^{\prime }\right)=\sum_{j=1}^{N}p\left(a_{k}\right)\left(a_{k}^{\prime }|a_{k}\right),\\ =p_{k}.p\left(a^{\prime }=s_{k}|a=s_{k}\right)+\theta \left(1-p_{k}\right). \end{array}$$

This can be measured assuming the *k*^th^ node of the application layer waiting to release its data with a segment connectivity of *s*_*k*_ with a suggested *j*^th^ service operator node of network layer.

## 5. Result Outcomes

We trained our system using five additional publicly available data sets from five different database servers. The connectivity included the government database through the referred website and the edge smart phone database as an edge server. We observe the consequence of our Hemayah model for different circumstances. We selected and observed a scenario of a public gathering with the help of a network-monitoring system [2]. This visualization is specifically based on java programming, which can generate an amazing graphical view of network activities. This GUI consists of packet request throughput, I/O, and captures packet flow along the connectors. We considered two scenarios; one without using the Hemayah application and the other using an existing application. With the help of the Hemayah application, the organization authority can connect with possible service as per the suggestion of QoS manager. Then we got two kinds of packet delivery activities in Figures 4 and 5.

RETRACTED

In Figure 4, the packet sending and delivery show that different mobile nodes use mobile operators and connect to a particular website to get information. This scenario is the same as Case 1 referred to in Section 3. In Figure 5 we can see the single authorized node (the entry point admin) scanning the physical status and updating latest information to the server against each individual, for further usage.

Compared one after another model with our proposed QoS-aware Hemayah model we come to the conclusion that our proposed model is more efficient in terms of packet failure, energy consumption of mobile phone battery, and delay over packet delivery than the other existing model.

Figure 6 depicts how the packet rate has suddenly increased when waiting in a queue and trying to access their data from an official site. In contrast, Figure 7 shows the I/O graph generated while using a single-point communication between the admin site of the entry point and the previously stored data at another authorized server. The second communication shown in Figure 7 is more reliable, time-efficient, data-efficient, and digitalized. The transmission is hassle-free, no need to bring hard copies of data or hand over the mobile phone to check your own local database.  Figure 8 depicts generated throughput graph for the connectivity from the checkpoint server to the HOM server for data checking, validation, and new scanning report upload. The communication occurs using single-point scanning and data checking and updating using Hemayah application.  Table 1 highlights a comparative analysis of our proposed solution with existing COVID-19 related models using Android-based applications.

## 6. Conclusion

Proposed Hemayah has potential as a multifunctional android-based application. Using visitor's National or Iqama ID, Hemayah allows users to check the status of anyone in front of them from their mobile phones without the need to use the visitor's phone. This feature contributed to Hemayah to overcome any problem that visitors face with their phones and thus not enabling them to access their current health status, as it happens in other applications [26, 27], which depends on showing the status of individuals through their phones. Another benefit of Hemayah is the Port Checkpoint where border point officials display PCR data (infected-uninfected). Displaying the traveler's PCR data will reduce the use of papers and ensure the reliability of the results because it was entered into the system through laboratories approved by Saudi authorities. The major efficiencies of proposed QoS-aware layered architecture at the backend of Hemayah app has been refined upon some aspects. Few of them are following:

- To make the Digital-based service more convenient while reducing possible physical contact.
- The reasonable service cost decreases; no need to carry a personal mobile phone for this particular task. Functioning effort on availability factors have been done efficiently.
- Some real time factors of android-based application nodes have been modified, like regularity, reliability; single node communication to increase robustness and reputation of the whole Hemayah network.

RETRACTED

As the training of the model highly depends upon the real-time data set, we can enhance the scope of our Hemayah model for the early prevention of similar pandemic crises. The only concern will be legal actions to reach an immense data set for thorough training. We believe our model has proved specific and highly reliable in every possible event. However, this article includes a few performance outcomes of our model in discussed circumstances. Furthermore, we are still trying to uplift the user experience or quality of experience (QoE) [28] in every possible aspect.

## Figures and Tables

**Figure 1:** Existing COVID-19 Android-based tracking and monitoring service flows of the proposed solution. (a) Request flow at the time of in-country service avail. (b) Request flow at the queues at border checkpoints.

**Figure 2:** Data flow diagram of the proposed three-layered architecture of the hemayah application.

**Figure 3:** Front end of the Hemayah: the statistics and last visited places details windows.

**Figure 4:** Packet request, send and received by individual mobile node within an existing network while using an indifferent app.

**Figure 5:** Packet request, send and received by authorized single node within an existing network while using a Hemayah app.

RETRACTED

**Figure 6:** Generated I/O graph while using different network operators by different mobile nodes and indifferent app.

**Figure 7:** Generated I/O graph while using single point scanning and data checking and update using Hemayah app.

**Figure 8:** Generated throughput graph while using single point scanning and data checking and update using Hemayah app.

**Algorithm 1:** QoS aware for Hemaya's database selection algorithm for iterative model.

**Table 1:** Comparison of proposed solution with existing COVID-19 related models using android-based applications.

Name of the application	Android-based user application	Distributed database for real-time learning	Considered QoS matrices	Service providing point of view	Data access procedure (one to one or many to one or many to many)
Sehhaty	Several health-related assistance	✓	✗	Multi service providing	Many source to one person
Mawid	E-Appointment app	✗	✗	Single serviced	Connects many hospitals to one
Tawakkalna	Helps to verify own health condition	✗	✗	Multi serviced	One to one
Tabaud	To track COVID-19 spread	✓	✓	Multi serviced	Many to one
Eshara	User specific, supports sign language	✓	✗	Multi serviced	Many to one
Qareboon	Offers text-based mental counselling	✗	✗	Multi serviced	Many to one
Hemayah (proposed)	Multi-user-based, helps to prevent pandemic outbreak	✓	✓	Multi serviced	Many to many

## Data Availability

The data used to support the findings of the study are included within the article.
